# The effect of a sports chiropractic manual therapy intervention on the prevention of back pain, hamstring and lower limb injuries in semi-elite Australian Rules footballers: a randomized controlled trial

**DOI:** 10.1186/1471-2474-11-64

**Published:** 2010-04-08

**Authors:** Wayne Hoskins, Henry Pollard

**Affiliations:** 1 Macquarie Injury Management Group, Department of Chiropractic, Faculty of Science, Macquarie University, NSW 2109, Australia

## Abstract

**Background:**

Hamstring injuries are the most common injury in Australian Rules football. It was the aims to investigate whether a sports chiropractic manual therapy intervention protocol provided in addition to the current best practice management could prevent the occurrence of and weeks missed due to hamstring and other lower-limb injuries at the semi-elite level of Australian football.

**Methods:**

Sixty male subjects were assessed for eligibility with 59 meeting entry requirements and randomly allocated to an intervention (n = 29) or control group (n = 30), being matched for age and hamstring injury history. Twenty-eight intervention and 29 control group participants completed the trial. Both groups received the current best practice medical and sports science management, which acted as the control. Additionally, the intervention group received a sports chiropractic intervention. Treatment for the intervention group was individually determined and could involve manipulation/mobilization and/or soft tissue therapies to the spine and extremity. Minimum scheduling was: 1 treatment per week for 6 weeks, 1 treatment per fortnight for 3 months, 1 treatment per month for the remainder of the season (3 months). The main outcome measure was an injury surveillance with a missed match injury definition.

**Results:**

After 24 matches there was no statistical significant difference between the groups for the incidence of hamstring injury (OR:0.116, 95% CI:0.013-1.019, p = 0.051) and primary non-contact knee injury (OR:0.116, 95% CI:0.013-1.019, p = 0.051). The difference for primary lower-limb muscle strains was significant (OR:0.097, 95%CI:0.011-0.839, p = 0.025). There was no significant difference for weeks missed due to hamstring injury (4 v14, χ2:1.12, p = 0.29) and lower-limb muscle strains (4 v 21, χ2:2.66, p = 0.10). A significant difference in weeks missed due to non-contact knee injury was noted (1 v 24, χ2:6.70, p = 0.01).

**Conclusions:**

This study demonstrated a trend towards lower limb injury prevention with a significant reduction in primary lower limb muscle strains and weeks missed due to non-contact knee injuries through the addition of a sports chiropractic intervention to the current best practice management.

**Trial registration:**

The study was registered with the Australian and New Zealand Clinical Trials Registry (ACTRN12608000533392).

## Background

Australian Rules football is a unique body contact sport. It is played on a natural grass, oval shaped field, with the size varying between 135 - 185 meters in length and 110 - 155 meters in width. Teams consist of 18 players per side plus four on an unlimited interchange bench. Each game is played over four 20 minute quarters plus stoppage time. Physical requirements of players include: repeated rapid acceleration and deceleration efforts often involving change of direction, agility, jumping, bending to pick up the oval shaped ball, tackling and other collisions [1]. There is a continuous nature of play requiring high aerobic capacity, although the speed of the game has increased and now involves a greater number of shorter high intensity play periods and longer stop periods [2]. The most important means of ball progression is by punt kicking. Australian Rules football has the highest rates of non-contact soft tissue injuries when compared with other body contact football codes such as rugby league and rugby union [3], with the incidence of lower limb muscle strains at the elite national competition, the Australian Football League (AFL), being 35% per season [4].

Hamstring injuries are the most prevalent injury in Australian Rules football at the AFL [4] and feature prominently at other levels of play [5]. Per season in the AFL hamstring injuries afflict 16% of players, cause 3.4 missed matches per injury, account for the most time missed due to injury and have the highest rates of injury recurrence, with one in three injuries recurring on return to play [4]. On return to play, player performance is significantly lower [6]. Hamstring injuries are also the most common muscle injury in running based sports [7]. Knowledge surrounding optimal preventative measures is therefore critical.

The prevention of hamstring injuries has long been recognized as a priority effort. By contrast, Bahr and Holme [8] have opined that well designed prospective hamstring injury prevention studies are lacking. Recent literature reviews have been universal in their depiction of the lack of evidence for the prevention of hamstring injuries and the requisite for evidence based approaches to be determined through randomized controlled trials (RCTs) [7,9,10]. Prevention of injury becomes more crucial as the most established predictors for hamstring injury in Australian Rules football are immutable in nature, namely a current or recent history of a hamstring injury and age [11].

Conventional injury prevention has focused on local hamstring factors. Orchard [11] has said that sports medicine dogma advises that poor flexibility, fatigue, lack of warm up and weakness are risk factors for injury. The evidence to support this tenet for hamstring injury is lacking [7]. However, a growing body of literature, largely of an indirect nature, suggests that several non-local hamstring factors may have an association with injury [12-16], whilst a Cochrane systematic review of the literature has stated that consideration should be given to the lumbar spine, sacroiliac and pelvic alignment and postural control mechanisms when managing hamstring injuries [17]. Despite the knowledge that non-local factors may exist, the literature appears almost devoid of research investigating their possible identification and documenting the effects, if any, of addressing non-local factors in hamstring injury management [12,16,18]. A recent review of the literature stated that newer approaches that incorporate manipulation in multi-modal management approaches for hamstring injury prevention should be further investigated [9]. Thus it was the objective of this RCT to investigate whether a sports chiropractic intervention consisting of pragmatically and individually determined high-velocity low-amplitude (HVLA) manipulation, mobilization and/or supporting soft tissue therapies to the spine, pelvis and extremity could reduce local and non-local hamstring injury risk factors to prevent the occurrence of hamstring and other non-contact lower limb injuries and decrease low back pain (LBP) and alter health outcomes in semi-elite Australian Rules footballers.

## Methods

### Protocol

Four of the thirteen clubs competing in the semi-elite state based Victorian Football League (VFL) were approached and agreed to provide players for this study during the 2005 season. However, a change in club staff resulted in two clubs withdrawing support prior to subject recruitment. VFL players train and play in the same competition as elite AFL players not selected for first grade competition and receive financial remuneration without being full time in their playing and training commitments. Players were eligible to participate if they were listed players on their respective VFL squad and excluded on the basis of: "red flag" conditions including: fractures, infections, inflammatory diseases, tumours and other causes of destructive lesions of the spine; "yellow flag" conditions including: insurance claims, litigation; history of malignant disease; clinical signs suggesting inguinal or femoral hernia; vascular disease; history of motor vehicle accident, or other serious fall or accident in the last three months; neurological signs and symptoms (muscle wasting, nerve root signs, bowel, bladder or sexual dysfunction); organic kidney, urinary tract or reproductive disease; previous recent spinal surgery (less than 2 years); club doctor or medical staff excludes the players participation; severe history of chronic hamstring problems; serious injury or surgery preventing play for the remainder of the season. Before the start of the study the subjects, coaches and medical personal were informed about the purpose and design of the study. Club staff gave permission to participate in the study.

### Assignment

Players completed a self-reported questionnaire at their training location prior to randomization. The questionnaire consisted of the validated and reliable McGill Pain Questionnaire (short form) (MPQ-SF) for LBP, the 39 item Health Status Questionnaire (SF-39) as well as self reported questions on knee and hamstring injury history (incidence during the previous month, 6 months, year, 2 years, greater than 2 years or not at all). At each of the two clubs after completion of the baseline questionnaire, players were randomly allocated into one of two groups such that allocation was concealed. Eligible players were stratified by age and hamstring injury history and allocated using a computer generated randomization list for each club within these strata, as these are the most recognized predictors for injury [11]. Randomization was completed within each club to prevent an element of randomness in a clubs injury profile each season impacting on the results of the study. After all subjects had been allocated the two groups at each club were then randomly allocated to either the intervention or control with a coin toss.

### Intervention

All of the players in both the intervention and control group continued to receive what is considered the current best practice medical, paramedical and sports science management including medication, manipulative physiotherapy, massage, strength and conditioning and rehabilitation as directed by club staff, which acted as the control. All treatment from club staff was independently administered without restriction or interference from the study authors. All staff were employed by the club and had no limitation in the number or type of treatment they could render. In addition to this, the intervention group received a sports chiropractic approach administered by a single practitioner. Treatment was pragmatically and individually determined by the therapist and could involve HVLA manipulation (either manual or mechanically assisted techniques), mobilization and/or supporting soft tissue therapies: various stretching and soft tissue massage techniques to the spine, pelvis and extremity. According to Mierau et al. [19] manual manipulation involves a brief, shallow, sudden carefully administered thrust (high velocity in nature). Mechanically assisted manipulation is performed through the assistance of devices (for example drop pieces) or impulse type instruments, being non-cavitational and high velocity in intent. Mobilization occurs when a joint is passively moved within its normal range of motion (usually a slow oscillatory movement). Treatment scheduling was also pragmatically determined. The minimum scheduling adhered to was: 1 treatment per week for 6 weeks (phase 1) followed by 1 treatment per fortnight for 3 months and 1 treatment per month for the remainder of the season (3 months) (phase 2).

### Outcome Measures

The study was divided into two phases. Phase 1 (6 weeks) involved the late pre-season period where pre-season matches and the intervention commenced but no injury surveillance was conducted. Phase 2 (24 weeks) occurred where regular season (home and away) and finals matches were conducted weekly and an injury surveillance was conducted. The injury surveillance commenced after a period of more intense treatment scheduling such that the treatment effects, if any, would be observed in a changed injury pattern. At the mid point of the season (12 home and away season matches, 18 weeks of intervention) players completed the MPQ-SF and the SF-39 as secondary outcome measures at their training location.

The injury definition and injury surveillance conducted was a reproduction of the AFL's injury surveillance and used as a primary outcome measure for the prevention of hamstring injuries, lower limb muscle strains and non-contact knee injuries [4]. The definition of an injury was: "any physical or medical condition that prevents a player from participating in a regular season (home and away) or finals match". The missed match injury definition is currently considered the most reliable injury surveillance method in team sports [20]. The number of games missed due to injury was also determined. Injury diagnoses were determined by club medical staff who were blinded to group allocation using either clinical features of injury, advanced imaging or both at their discretion with blinded club recorders completing the injury surveillance. Clinical parameters of injury were also recorded including mechanism of injury (contact or non-contact). In this way separation of injuries could be made retrospectively and allocated into groups for statistical analysis. To attain this, the player was interviewed at the first available opportunity following injury. The club medical and coaching staff independently determined selection in matches. There was no interference from the study authors.

In addition a secondary injury surveillance for adverse outcomes resulting from the intervention was established for the duration of the study with an injury definition of: "any undue pain, discomfort or disability arising during, immediately after or subsequent to chiropractic therapy that resulted in missed participation in a match or training session, required additional medical consultation or treatment or was acknowledged by a player as not reasonably being associated or expected with the normal course of treatment". If an injury occurred, further details on the type of injury, timing of symptom onset, duration of symptoms and severity were to be determined.

### Statistical Analysis

All data collected were manually entered using Microsoft Excel and analyzed using SPSS for Windows (version 12.0) or for weeks missed due to injury, SAS version 9.1.3 and PROC GENMOD. Pearson's "exact" Chi-squared test based on Monte Carlo simulation was used to assess the efficacy of the intervention with respect to the number of injuries. Odds ratios and 95% confidence intervals were also included. As such this calculation is just an approximation and is included as it is believed that confidence intervals should always be stated [21]. Negative binomial models were used to calculate significance for weeks missed due to injury. Two independent sample t-tests were used to compare group age, hamstring and knee injury history, MPQ-SF and SF-39 at baseline, or if distributions were mixed, Fisher's exact test was used. Repeated measures and regression models were used to determine change for the MPQ-SF and SF-39. If data were extremely skewed in distribution, transformation of scores was required. Between group differences were obtained from two independent sample t-tests. For global statistical tests, a p value < 0.05 was considered significant.

### Statistical power calculation

Based on historical AFL data [4] the assumed hamstring incidence level for the null hypothesis is 15%. For a 5% significance level and 80% power, a total sample size of 117 is required to detect a 50% reduction in the incidence of hamstring injuries.

### Ethical considerations

All players gave their written informed consent to participate and ethical approval was obtained from the Macquarie University Human Ethics Committee (Ethics Approval Number: HE27AUG2004-RO3066).

## Results

### Participants

Sixty male Australian Rules football players were recruited as subjects. Figure 1 shows a flow chart describing progress of subjects through the trial for the primary and secondary outcome measures. Players were randomly allocated to the intervention (n = 29) or control group (n = 30) with no baseline differences for age (mean/SD/range intervention 20.2/1.8/18-27, control 20.2/1.8/18-25), self-reported hamstring and knee injury history, MPQ-SF and SF-39 (all p > 0.05).

**Figure 1:** **CONSORT flow chart indicating progress of subjects through the trial**.

### Injury Surveillance

Table 1 presents the results for the difference in injury incidence between the groups at the completion of the season (24 matches, 30 weeks of intervention). There was no statistical difference in the prevention of hamstring injuries (p = 0.051) or weeks missed due to hamstring injury (χ^2 ^1.12, p = 0.29). For primary hamstring injuries, the incidence was 3.6% for the intervention group and 17.2% for the control group, with the recurrence rate being 40.0%. The intervention group missed 4 matches due to hamstring injury and the control 14 matches. The intervention group was at a statistically significant reduced risk of suffering a primary lower limb muscle strain injury (p = 0.025), equating to 3.6% of the intervention group and 27.6% of the control group. The intervention group missed 4 matches with a lower limb muscle strain and the control group 21 matches (χ^2 ^2.66, p = 0.10). The difference in primary non-contact knee injury incidence was not statistically significant (p = 0.051), with the incidence being 3.6% for the intervention group and 24.1% for the control group. The intervention group missed 1 match with a primary non-contact knee injury and the control group 24 matches, the difference being statistically significant (χ^2 ^6.70, p = 0.01). No players reported an adverse reaction to the intervention.

**Table 1:** Difference between the intervention and control group for injury incidence at the completion of the season (24 matches, 30 weeks of intervention)

Injury	Intervention incidence (n = 28)	Control incidence (n = 29)	P value	Odds ratio	95% CI
Hamstring injury	1	7	0.051	0.116	0.013-1.019

1° Hamstring	1	5	0.191	0.178	0.019-1.631

2° Hamstring	0	2	-	-	-

**1° Lower limb muscle strain**	1	8	0.025*	0.097	0.011-0.839

1° Non-contact knee	1	7	0.051	0.116	0.013-1.019

* Bold type face indicates significant difference

### Low Back Pain

Table 2 presents the results for the change in baseline MPQ-SF at the mid point of the season. A positive and statistical significant change for the intervention group was achieved for overall (p = 0.006) and current LBP (p = 0.026). No significant change was noted for the other components of the MPQ-SF (p > 0.05).

**Table 2:** Lower Back Pain (as measured by the MPQ-SF): estimated marginal means for baseline and eighteen weeks by group and estimated change within and between groups

Variable		Baseline		18 weeks		Δ within groups		Δ between groups	
		**intervention**	**control**	**intervention**	**control**	**intervention**	**control**	**mean**	**p-value**

**Current**	mean	33.26	32.71	21.44	34.36	-11.81	1.64	-13.46	**.026**

	*95% CI*	*24.00, 42.52*	*23.62, 41.81*	*12.77, 30.12*	*25.84, 42.88*	-*22.90, -0.73*	-*8.8, 12.14*	-*28.35, 1.44*	

**Overall**	mean	26.67	22.86	17.04	27.86	-9.63	5.00	-14.63	**.006**

	*95% CI*	*20.54, 32.80*	*16.84, 28.88*	*10.67, 23.41*	*21.60, 34.11*	-*16.35, -2.91*	-*3.07, 13.07*	-*24.93, -4.33*	(.034)^1^

Sensory	mean	12.57	15.26	13.02	18.20	0.45	2.94	-2.49	.461

	*95% CI*	*8.56, 16.59*	*11.32, 19.20*	*8.02, 18.03*	*13.29, 23.11*	-*3.67, 4.57*	-*2.54, 8.43*	-*9.24, 4.25*	

Affective	mean	4.95	4.76	8.33	10.72	3.38	5.96	-2.58	.411

	*95% CI*	*1.78, 8.12*	*1.65, 7.87*	*3.96, 12.70*	*6.43, 15.01*	-*0.73, 7.48*	*1.07, 10.85*	-*8.84, 3.6*	

Total	mean	10.53	12.56	11.81	16.19	1.28	3.63	-2.35	.436

	*95% CI*	*7.0, 14.06*	*9.10, 16.02*	*7.24, 16.38*	*11.70, 20.67*	-*2.57, 5.12*	-*1.14, 8.40*	-*8.36, 3.66*	

* Bold type face indicates significant difference between groups at 18 weeks.

1 Regression analysis showed a significant difference between groups: p-value calculated using regression analysis.

### Health Status

Table 3 presents the results for the change in baseline SF-39 at the mid point of the season. A positive statistical change for the intervention group was achieved for role limitations due to physical health (p = 0.004), bodily pain (p = 0.034), general health (p = 0.027), and physical summary score (p = 0.013). No other statistically significant change was noted for other health status components (p > 0.05).

**Table 3:** Health status (as measure by the SF-39): estimated marginal means for baseline and eighteen weeks by group and estimated change within and between groups

Variable		Baseline		18 weeks		Δ within groups		Δ between groups	
		**intervention**	**control**	**intervention**	**control**	**intervention**	**control**	**mean**	**p-value**

Physical functioning	% at 100	65.50	60.00	55.60	33.30	-2.41^2^	-4.26^2^	1.85^2^	.569

	*95%CI*	*48.20, 82.80*	*42.47, 77.53*	*36.86, 74.34*	*15.52, 51.08*	-*5.72, 0.90*	-*11.59, 3.07*	-*6.08, 9.79*	

**Role limitation-physical**	% at 100	72.40	80.00	85.20	40.70	9.26^2^	-18.52^2^	27.78^2^	**.004**

	*95%CI*	*56.13, 88.67*	*65.69, 94.31*	*71.81, 98.59*	*22.17, 59.23*	-*2.43, 20.94*	-*31.84, -5.20*	*10.48, 45.08*	

**Bodily pain**	Mean	69.67	72.56	74.22	65.26	4.56	-7.30	11.85	**.034**

	*95%CI*	*63.68, 75.66*	*66.57, 78.55*	*67.43, 81.01*	*58.47, 72.05*	-*4.09, 13.21*	-*14.36, -0.24*	*0.95, 22.75*	

**General health**	Mean	81.30	79.00	83.96	74.52	2.67	-4.48	7.15	**.027**

	*95%CI*	*76.51, 86.08*	*74.22, 83.78*	*78.51, 89.42*	*69.06, 79.97*	-*2.53, 7.86*	-*10.27, 1.31*	-*0.45, 14.74*	

Vitality	Mean	60.37	61.11	67.04	59.44	6.67	-1.67	8.33	.050

	*95%CI*	*53.90, 66.84*	*54.64, 67.59*	*61.67, 72.40*	*54.08, 64.81*	-*0.57, 13.90*	-*9.15, 5.81*	-*1.83, 18.49*	

Social functioning	% at 100	51.70	53.30	58.10	44.40	0.46^2^	-5.09^2^	5.56^2^	.770

	*95%CI*	*33.51, 69.89*	*35.45, 71.15*	*39.49, 76.71*	*25.66, 63.14*	-*4.76, 5.68*	-*11.56, 1.38*	-*2.56, 13.67*	

Role limitation-emotional	% at 100	75.90	83.30	92.60	66.70	8.64^2^	-6.17^2^	14.81^2^	.142

	*95%CI*	*60.33, 91.47*	*69.95, 96.65*	*82.73, 102.47*	*48.92, 84.48*	-*0.75, 18.03*	-*16.54, 4.20*	*1.16, 28.47*	

Mental health	Mean	77.63	77.93	76.59	71.11	-1.04	-6.81	5.78	.151

	*95%CI*	*72.50, 82.76*	*72.80, 83.06*	*71.61, 81.57*	*66.13, 76.09*	-*6.60, 4.52*	-*12.78, -0.85*	-*2.18, 13.74*	

**Physical summary score**	Mean	52.66	52.03	53.80	49.06	1.15	-2.97	4.12	**.013**

	*95%CI*	*50.63, 54.68*	*50.00, 54.06*	*51.76, 55.85*	*47.01, 51.10*	-*1.14, 3.43*	-*5.36, -0.58*	*0.89, 7.35*	

Mental summary score	Mean	50.04	50.55	51.41	48.48	1.37	-2.07	3.45	.103

	*95%CI*	*47.21, 52.87*	*47.72, 53.38*	*49.00, 53.83*	*46.06, 50.89*	-*1.38, 4.12*	-*5.34, 1.19*	-*0.72, 7.61*	

Depression	% at 100	58.60	73.30	85.20	59.30	9.89^2^	-3.70^2^	13.59^2^	.050

	*95%CI*	*40.67, 76.53*	*57.47, 89.13*	*71.81, 98.59*	*40.77, 77.83*	*1.87, 17.90*	-*12.15, 4.74*	*2.23, 24.96*	

* Bold type face indicates significant difference between groups at 18 weeks.

### Intervention

Table 4 provides a description of the treatment rendered to the intervention group for the course of the study.

**Table 4:** Description of the treatment rendered to the intervention group

	Intervention group (n = 29)
Number of treatments	487 (mean per player 17)

Amount of manipulation and/or mobilization to joint regions	2000 (47% total treatment, mean 4 per treatment)

Location of manipulation and/or mobilization	Thoracic spine 21%, knee 18%, hip 18%, lumbar spine 15%, sacroiliac joint 12%

Manipulation and mobilization breakdown	HVLA manipulation only 56%, HVLA manipulation and mobilization 36%, Mobilization only 8%

Amount of soft tissue techniques to soft tissue regions	2258 (53% total treatment, mean 4 per treatment)

Location of soft tissue techniques	Gluteal region 22%, lumbar spine 12%, hip flexors 10%, knee 9%, posterior thigh 6%

* Soft tissue structures are defined as surrounding the involved joint (muscle, tendon, ligament, fascia etc.)

## Discussion

This RCT demonstrated that a sports chiropractic manual therapy intervention provided at the semi-elite level of Australian Rules football in addition to the current best practice multi-disciplinary medical, paramedical and sports science management resulted in the prevention of primary lower limb muscle strain injuries, although no statistical significance was noted for hamstring injury and primary non-contact knee injury. The addition of the intervention was associated with a reduced number of matches missed due primary non-contact knee injury, although no statistical significance was noted for hamstring injury and primary lower limb muscle strains. In addition, reduction in LBP was observed along with improvements in some aspects of the physical components of health status as measured by the SF-39. Treatment was predominantly directed at non-local to hamstring areas, which supports the view that several non-local factors may potentially contribute to hamstring and lower limb injury occurrence [7,9], which may be addressed through multimodal and multidisciplinary management [16]. These findings are important due to their potential for injury reduction, performance benefit and cost saving practices for a relatively low cost intervention.

There are limitations in the presented study. Because the required subject numbers as determined by the power analysis was not achieved, care is needed in the interpretation of the results. The late withdrawal of two clubs reduced the subject numbers recruited and meant that the required target of subject numbers would not be reached. Due to the late withdrawal it was decided to continue with the study. However, the number of subjects determined by the power analysis is based on an arbitrary determined effect size, and the numbers required would have been different if another effect size had been chosen. Moreover, the results that are presented report statistical significance and it is difficult to determine what difference in the raw figures would be clinically significant. As the level of significance for prevention of hamstring injuries and primary non-contact knee injuries was p = 0.051, given that the study was short of the number of subjects required by the power analysis, there is a strong likelihood of a type 2 error, especially considering how close each of these results were to p < 0.05. With regards to the fact that lower limb muscle strain injury incidence was significantly lower while the missed weeks was not, this implies that many minor grade strain injuries may have been prevented, but the one injury causing 4 missed matches skewed the results and meant the comparison would not be statistically significant. This is important in a small sample study such as the prevention of one serious injury (or not) can significantly alter the weeks lost profile of a particular treatment approach. Only studies with much larger sample sizes can really effectively confirm this important research observation.

Furthermore, a question could be raised regarding control group selection. It was felt that using the club based best practice medical, paramedical and sports science management as the control was valid because no change in hamstring injury rates using this same approach have been documented in the AFL's long running injury surveillance [4]. Corroborating this viewpoint, the hamstring injury incidence reported for the control group (17%) was very similar to that reported in AFL players (16%) using the same methodology. Difficulty arises in attempting to perform research on high-level professional or semi-professional athletes due to clubs not being overly enthusiastic for researchers to perform interventions on their contracted and paid players, particularly if the intervention to be performed is purely for control purposes. To counter this dilemma a pragmatic approach to research design was taken which created a further limitation in that subjects were not blinded to group allocation, meaning it cannot be ruled out that the intervention effect was due purely to placebo or Hawthorne effects, particularly as there was no blinding of the therapist. However, more modern research design often requires new interventions to be compared with the existing best practice approach [22], which was done in this study.

The injury surveillance for adverse reactions to treatment may be limited due to the subjectivity of aspects of the injury definition. Players may not have self-reported injury. If injury was delayed or transient, players may not have attributed injury to the intervention, instead attributing it to training/competition activities or other medical, paramedical or sports science management. Such a problem exists in any multi-modal management scenario. Conversely, given the reliability of the missed match injury definition [20], it is highly unlikely that a more severe injury resulting in loss of competition match play was missed.

The diagnosis of hamstring strains is usually made on clinical grounds [23]. Hamstring strains are commonly diagnosed through history (acute onset, non-contact mechanism) and examination (local tenderness, reproducible pain on straight leg raise testing and/or resisted knee flexion) [24]. In professional sport, MRI assessment is often used to support the clinical diagnosis and provide further assessment of the extent and severity of the injury. However, costs and availability preclude the use of this modality for routine assessment outside of professional sport. Additionally, both clinical examination and MRI findings are strongly correlated with the time required to return to competition, suggesting MRI is not required for estimating the duration of rehabilitation of an acute minor or moderate hamstring injury [25]. MRI imaging to confirm diagnosis of hamstring strains was not routinely performed in this study. There are limitations in relying on both clinical methods of diagnosis and MRI as hamstring injuries can appear clinically but not on MRI and they also may appear on MRI but not clinically [25]. As MRI was not routinely used, there is a possibility that some of the hamstring injuries in this study may have been MRI negative which are often considered "back related". There is some controversy regarding "back related" hamstring injuries as to whether a muscle strain is the cause, particularly for minor strains where causes for the pain may include referred pain from neuromeningeal or myofascial structures such as the lumbar spine and sciatic nerve or from nearby muscles such as the gluteal and pirifomis [23]. However, "back related" hamstring injury is an undefined term generally signifying both local hamstring signs and positive lumbar signs [23]. It should be noted that none of the hamstring injuries in the study had positive lumbar signs present at the time of diagnosis, but the lack of MRI diagnosis remains as a limitation of the study.

The intervention applied in this study was based largely on indirect evidence and speculative reasoning that local and non-local factors could potentially contribute to hamstring injury, which have been suggested to act as a guide to a complete prevention program [9]. Similar hypotheses could be made regarding other lower limb muscle strain injuries and non-contact knee injuries. As a uni-modal approach was not adopted to address a single risk factor, it is unclear as to what the specific mechanism of improvement was or what component of the protocol resulted in injury prevention. The multi-modal intervention was decided upon on the basis that it more accurately represents sports chiropractic clinical practice [26-28], and because sports injuries, including hamstring injuries, result from a complex interaction of multiple risk factors and events, of which only a fraction have been identified [8]. For the reversible risk factors that exist for hamstring injury, no definitive evidence exists to support them [7]. It has been suggested that waiting for a substantial body of evidence to exist to support a risk factor in its role in injury before conducting a RCT may be considered unethical [8].

Whilst a multi-modal approach was adopted, we speculate that the most significant difference between the control and the intervention groups was the inclusion of a significant amount of HVLA manipulation, as soft tissue therapies were habitually administered to the athletes in this cohort. Although data were not recorded in this study, manipulation if used by manipulative physiotherapists (as in the control group) has a tendency to be slow velocity or mobilization in nature and if HVLA techniques are rendered they are characteristically done so sparingly [29]. In the paper by Flynn et al. [29] they state that in the previously reported low back pain literature high velocity spinal manipulation utilization rates for low back pain to be between 2.8% and 8.9%, with rates in a heavily evidence based education system to be 36.2%. Alternatively, in the cited studies low velocity mobilization is used between 27.2% and 72.0% of the time. Despite these figures being the most up to date yet published, these figures represent United States, Ireland and United Kingdom physiotherapists and the figures may not be representative of current practice in those geographical locations or in Australian physiotherapists in particular. In contrast, the sports chiropractic intervention provided to the intervention group had a greater emphasis on performing HVLA manipulative techniques to both spinal and extremity joints, with 92% of total joint based treatment involving some form of HVLA manipulation technique. Future research would benefit from recording the nature of the control interventions in order to clarify the differences between interventions or to specifically address the role of HVLA based manipulative techniques. Future studies could specifically document the scope of the manual treatment delivered by all treating practitioners in both groups, which would assist in comparing outcomes. A criticism of manual therapy interventions is that its effects are short term in nature. Because of this, it was decided that an ongoing treatment approach with adequate spacing of treatments during the season would be applied. This would also best manage ongoing injury and sub-clinical micro-trauma or gradual onset injury that could occur to players over the course of the season. The decision on the minimum scheduling of treatment decided upon for the intervention group was made such that there would be a likely treatment effect. Treatment scheduling in this pragmatic arrangement was then based upon current and previous player medical history, examination findings, practicality, player preference and practitioner experience. As the intervention was provided by a single practitioner, this removed issues associated with inter-practitioner reliability. As mentioned in the results there was an average of 17 treatment consultations administered per player in the intervention group, but due to the pragmatic nature of the design, not all players received the same amount of treatment.

Sherry and Best [18] have suggested that neuromuscular control of the lumbopelvic region is needed to create optimal function of the hamstrings. They further suggest that changes in neuromuscular control could lead to changes in length tension relationships or force-velocity relationships of the hamstrings, predisposing injury. This hypothesis could extend to other muscle groups including quadriceps and groin muscles. Other authors have also hypothesized that dysfunction of the axial skeleton may predispose abnormal hamstring functioning that may relate to a greater incidence of injuries [7,9,16], which is supported by evidence documenting lumbopelvic factors as risk factors for hamstring injury [12-15]. Supporting this mechanism of injury is the large body of literature showing that LBP is associated with changes in lumbopelvic muscle activation and recruitment [30,31], including early activation of biceps femoris and alteration in neuromuscular control strategies [32], all of which could contribute to injury. In athletes, changes in lumbopelvic stabilization exist following clinical recovery of LBP [33]. Noteworthy is the high prevalence, frequency and severity of LBP occurring in the subjects recruited for this study [34].

Although the neurophysiological mechanisms underlying HVLA manipulation are not fully known or understood [35], evidence exists showing it is capable of stimulating muscle spindles, pacinian corpuscles and golgi tendon organs greater than that achieved by slow velocity mobilization [36]. Panjabi [37] has hypothesized that injured spinal mechanoreceptors may alter afferent input, effecting motor unit recruitment. Alterations in the recruitment of motor units of the deep lumbopelvic muscles may result in altered lumbopelvic stabilization strategies and insufficient force generated by the hamstrings and other muscles attached to the pelvis, or may result in excessive force production, causing subsequent injury. Alterations in hamstring motor units may also occur. Stimulation of mechanoreceptors by HVLA manipulation may improve afferent feedback required to update and modify motor functions. This may improve neuromuscular control of the lumbopelvic region and/or the coordination of hamstring and pelvic muscle function, preventing injury. In support of such a view, Solomonow et al. [38] have demonstrated that discharge of spinal proprioception can produce change in multifidus activation. Additionally, HVLA spinal manipulation has been shown to produce significant improvements in feed forward activation times of deep abdominal musculature [39], whilst case reports have shown it may improve the ability to perform transversus abdominus [40] and multifidus contraction [41]. Collectively these deficiencies have been found to be associated with LBP, with transverses abdominus and multifidus being key stabilizers in lumbopelvic stabilization [30,42]. Studies have also indicated that HVLA manipulation may improve muscle function through either facilitation or disinhibition of neural pathways [35]. These effects, combined with spinal manipulation improving hamstring strength [12], and increased joint mobility through mechanical stretching and neurophysiological mechanisms [35], may have lead to improvements in hamstring and other lower limb muscle functioning and subsequent injury prevention noted in this study. Due to the complex multi-factorial etiology underlying hamstring and lower limb muscle injury, it is probable that more than one possibly interacting mechanism occurred to prevent injury. Additionally, the targeted inclusion of soft tissue therapies and extremity joint mobilization and manipulation stretching soft tissues and improving joint mobility may have potentially contributed to injury prevention.

The trend towards reduction in primary non-contact knee injuries and significant improvements in weeks missed due to these injuries may appear surprising. However, recent literature has documented the more precise details of the biceps femoris anatomy, which have not previously been appreciated [43]. The authors hypothesized that there may be a synergistic effect between biceps femoris and popliteus, signifying bicep femoris' important role in knee joint stabilization [43]. This may highlight the important bidirectional inter-play between hamstring and knee function. Thus, soft tissue treatments delivered to the popliteus and knee region and HVLA manipulation to the knee may have assisted with knee function and therefore led to prevention of knee injury. Lastly, research has shown that HVLA spinal manipulation can reduce knee extensor inhibition associated with anterior knee pain [44], which could lead to improvements in knee function and injury prevention. Of interest, LBP has also been associated with inhibition of the knee extensor muscles [45], which could imply a link between lumbopelvic and knee function. The potential role of the knee in hamstring injury has been discussed elsewhere in further detail [7].

Due to constraints in manuscript size, we are unable to describe the entire treatment provided in this study or to speculate on all proposed mechanisms of improvement, which will be the subject of a subsequent publication. It should be noted that treatment provided was patient specific and addressed both kinetic and kinematic chain variables. The treatment was representative of the 'modern multimodal' (MMM) chiropractic approach that has been described in the sports chiropractic literature [26,27], and recommended in selecting a chiropractor for the management of athletic injuries [28].

## Conclusions

Based on the limitations of this study which includes a low sample size, this RCT demonstrated that a sports chiropractic intervention comprising significant amounts of HVLA manipulation and soft tissue therapies provided in addition to the current best practice medical, paramedical and sports science management appears to be beneficial for the prevention of lower limb muscle strain injuries, weeks missed due to primary non-contact knee injuries and reduction of LBP and improvement in physical components of health status. In addition, although not statistically significant, there was a trend towards prevention of hamstring and primary non-contact knee injuries and there were no reported adverse outcomes from the intervention. The interesting trend in results but non-statistically significance should be replicated using a larger sample size to remove the short comings of this study. Based on the findings of this study due consideration should be given for the inclusion of sports chiropractic in the management options of elite athletes.

## Competing interests

The authors declare that they have no competing interests.

## Authors' contributions

WH and HP conceived the idea of the study. WH performed recruitment of subjects, data entry and the intervention. WH and HP contributed to writing draft documents and the final manuscript. Both authors read and approved the final manuscript.

## Pre-publication history

The pre-publication history for this paper can be accessed here:

http://www.biomedcentral.com/1471-2474/11/64/prepub
